The article "ORMDL3 Promotes Angiogenesis in Chronic Asthma Through the ERK1/2/VEGF/MMP-9 Pathway" was retracted in 2025. Reasons: unreliable data; unreliable results or conclusions; concerns about the data.

# ORMDL3 Promotes Angiogenesis in Chronic Asthma Through the ERK1/2/VEGF/MMP-9 Pathway

**DOI:** 10.3389/fped.2021.708555

**Published:** 2022-02-16

**Authors:** Zhen Ding, Fei Yu, Yan Sun, Ning Jiao, Lina Shi, Jinghong Wan, Qinghua Liu

**Affiliations:** ^1^Department of Pediatrics, Zibo Hospital of Traditional Chinese Medicine, Zibo, China; ^2^Department of Pediatrics, Shandong Provincial Hospital Affiliated to Shandong First Medical University, Jinan, China

**Keywords:** ORMDL3, angiogenesis, asthma, VEGF, MMP-9, ORMDL sphingolipid biosynthesis regulator 3

## Abstract

**Aim:**

Angiogenesis plays a vital role in airway remodeling in chronic asthma. ORMDL3 has been identified to be closely associated with the development of asthma remodeling. This study was to investigate the mechanism of ORMDL3 in angiogenesis of chronic asthma.

**Methods:**

BALB/c mice were divided into three groups, including an asthmatic group (group A), a budesonide-treated group (group B), and a normal control group (group C). Hematoxylin and eosin and Masson staining were used to evaluate the pathological changes. Angiogenesis in lung tissue was examined by CD31 staining. The changes of ORMDL3, ERK1/2, and angiogenesis-associated MMP-9 and Vascular endothelial growth factor (VEGF) expression were examined. Furthermore, ORMDL3, MMP-9, and VEGF mRNA and protein levels were examined after transfection in BEAS-2B cells with the ORMDL3-overexpressed lentiviral vector.

**Results:**

Compared with the control group, asthmatic mice indicated more severe airway angiogenesis with increased ORMDL3, ERK1/2, MMP-9, and VEGF expression. Budesonide alleviated airway angiogenesis, and CD31 expression was positive with the levels of ORMDL3, MMP-9, and VEGF (*P* < 0.01). After successful transfection in BEAS-2B cells with the ORMDL3-overexpressing lentiviral vector, VEGF, and MMP-9 expression were activated *in vitro* (*P* < 0.01).

**Conclusion:**

In conclusion, our study provides novel evidence that ORMDL3 promotes angiogenesis through upregulating VEGF and MMP-9 in chronic asthma.

## Highlights

- To investigate the potential influences of ORMDL3, we examined the expression of ORMDL3, ERK1/2, CD31, VEGF, and MMP-9 in OVA-stimulated BALB/c mice using immunohistochemistry, RT-PCR, and Western blotting in 12 weeks. And we found that ORMDL3 expression was greatly increased in the model group compared with the treated group and control group in 12 weeks, which had a significant correlation with VEGF, MMP-9, CD31 expression, and activated ERK levels.
- Budesonide could alleviate airway remodeling, which might due to inhibition of ORMDL3, VEGF, CD31, MMP-9, and ERK levels. Angiogenesis in lung tissue was examined by CD31staining. The expressions of ORMDL3, ERK1/2, MMP-9, and VEGF were examined through immunohistochemistry, RT-PCR, and Western blotting respectively.
- To investigate the expression and localization of ORMDL3 in asthmatic lung tissue, and to explore the effect of ORMDL3 and the molecular biological mechanism of angiogenesis in asthma remodeling in OVA-stimulated BALB/c mice using immunohistochemistry, RT-PCR, and Western blotting in 12 weeks. The effects of ORMDL3/ERK1/2/VEGF/MMP-9 on vascular remodeling in asthmatic mice were evaluated.
- The overexpression of ORMDL3 significantly increased after infection cells with lentiviral vector. Furthermore, MMP-9 and VEGF levels were examined by PCR after the transfection of BEAS-2B cells with the ORMDL-overexpressed lentiviral vector, which indicated that ORMDL3 overexpression induced activated expression of VEGF and MMP-9 *in-vitro*.
- The effects of ORMDL3/ERK1/2/VEGF/MMP-9 on vascular remodeling *in-vitro* were evaluated.

## Introduction

Over the past 20 years, asthma has been a major global public health concern, and the incidence rate has doubled with a younger age trend, the estimated prevalence of which is reported in different countries: 10% in the United Kingdom, 4.8% in France, and 4.8% in Germany approximately (1, 2). Asthma is a chronic airway inflammation characterized by airway hyperresponsiveness and remodeling. Angiogenesis, namely, the increase in size and number of blood vessels in asthma, increases the thickness of the airway wall and exudation of inflammatory factors (3). Angiogenesis in the bronchial airway results in more serious chronic inflammation because a well-developed network of blood vessels enables migration of inflammatory cells into the bronchial wall, which results in bronchial airway remodeling.

This study is devoted to investigating the functions and mechanisms of individual genes in angiogenesis in asthma. To date, ORMDL3 has been found to be strongly linked to asthma (4). Elevated ORMDL3 expression is detected in more than one-third of asthmatic children younger than 7 years of age. Chen et al. found that ORMDL3 regulated airway smooth muscle hyperplasia, airway smooth muscle contraction, and Ca^2+^ oscillations in asthma (5). ORMDL3 also contributes to the occurrence and development of airway remodeling and bronchial epithelial-mesenchyme transition (EMT) in asthma (6). However, the direct evidence of a relationship between the angiogenesis and ORMDL3 in asthma has not been fully elucidated. Vascular endothelial growth factor (VEGF) and matrix metalloproteinase-9 (MMP-9) are the important angiogenesis-promoting cytokines in asthma (6–8). The expressions of these factors are to be explored, and further works are severely needed to figure out the mechanisms of ORMDL3 in chronic asthma angiogenesis.

## Materials and Methods

### Animals

A total of 45 male BALB/c female mice (6 weeks) were bought from the experimental animal center of Shandong University (Jinan, China). The mice were maintained in an animal center under standard laboratory conditions. All mouse experiments accorded with the guidelines of Shandong University for the use of laboratory animals, and all measures were taken to keep animal suffering to a minimum.

### Murine Model of Asthmatic

The murine chronic model of asthma was established as previously described (8). All mice were randomly divided into three groups as follows (*n* = 15): asthmatic group (A), budesonide-treated group (B), and normal control group (C). Mice for groups A and B were sensitized on days 1, 7, and 14 by intraperitoneal (ip.) injection of the mixture of 100 ug OVA (Grade V, Sigma, U.S.) and 1 mg aluminum hydroxide (Aldrich, Milwaukee, WI) diluted in phosphate-buffered saline (PBS). Then, they were challenged with 1% OVA three times per week for 30 min from day 28 for groups A and B. Mice in group B were administered 30-min aerosol budesonide (Astra Zeneca, Lund, Sweden) (100 μg/kg) three times per week from day 21 before each OVA challenge. Mice in group C were sensitized and challenged with PBS instead. Aerosol budesonide was treated using a Germany Berry nebulizer (Inqua Neb PLUS). Twelve weeks later, all the mice were anesthetized and sacrificed after the last challenge.

### Hematoxylin and Eosin Staining

The lungs were collected, and tissue sections were prepared. Five-micrometer sections were stained with hematoxylin and eosin (HE), each specimen with a complete tracheal cross was observed via microscope (Leica, DM4000B). The indices of peribronchial inflammation were determined according to the following histological grading system: level 1:? 5% inflammatory cells, level 2: 5–25% inflammatory cells, level 3: 25–75% inflammatory cells, level 4: one definite layer of peribronchial inflammatory cells completely surrounding a bronchus, level 5: two definite layers of peribronchial inflammatory cells completely surrounding a bronchus, level 6: three or more layers of peribronchial inflammatory cells surrounding a bronchus. Inflammatory degrees in each group were calculated (8–10).

### Masson Staining

The Masson staining sections were quantitated to estimate the extent of collagen fiber deposition in asthma (10, 11). Four level scores were determined according to the collagen staining area: level 0:? 5%, level 1: 5–25%, level 2: 25–75%, and level 3:? 75% filamentous collagen. Five high-powered fields of each specimen were reviewed in a random blinded field by two independent investigators.

### Immunohistochemistry

Expressions of ORMDL3, MMP-9, p-ERK, VEGF, and CD31 in lung tissues were assessed by immunohistochemical staining. Samples were incubated with antibodies directed to ORMDL3 (Abcam, 107639), p-ERK (CST 4370), MMP-9 (Millipore, AB19016), VEGF (Millipore, ABS82), and CD31 (Abcam, ab28364) overnight, respectively. Then, samples were detected with biotinylated secondary antibodies and SAB reagent (Beijing Chinese fir Jinqiao). Five fields of each specimen were reviewed, and samples were assessed using Image J software.

### Western Blotting

Lung tissue protein was determined though a Bio-Rad protein assay, to which proteinase inhibitors were added. Forty microgram tissues of lung were loaded on to an SDS-PAGE with antibodies directed to ORMDL3 (molecular weight: 17 kDa Abcam107639, 1:1,000), ERK (molecular weight: 42 kDa, CST 9102, 1:1,000), p-ERK (molecular weight: 44 kDa, CST 4370, 1:1,000), MMP-9 (molecular weight: 92 kDa, Millipore AB19016, 1:1,000), and GAPDH (1:2,000).

### Infection of BEAS-2B Cells by Lentiviral Vector

The linearization vector was obtained by restriction enzyme digestion. The recombinant product was identified by PCR. High-purity plasmids were obtained from the expanded culture and extraction of the correct clone liquid. The mixture was slowly added to cell culture medium, mixed, and cultured. The fluorescence rate was the positive infection rate.

### Detection of ORMDL3, MMP-9, and VEGF With Western Blotting and RT-qPCR

The stably infected cells were incubated with the linearization vector. The sensitized cell monolayers were stimulated by lentivirus before two washes with RIPA lysis buffer; Western blotting analyses were performed as described previously: ORMDL3, VEGF (1:2,000), MMP-9 (1:500), and β-actin (1:10,000).

Cells were collected (80% cell density) using TRIzol reagent (Pufei, China), and mRNA was transcribed into cDNA using the PrimeScript RT Master Mix Perfect Real-Time kit (Takara Biotechnology Co., Ltd., Dalian, China). RT-PCR was performed using cDNA and SYBR-Green (Takara Biotechnology Co, Ltd). Expression levels of ORMDL3, MMP-9, and VEGF were normalized to GAPDH. The primers for RT-qPCR were given in Table 1.

**Table 1:** The primers used to detect ORMDL3, GAPDH, MMP9, and VEGF expression.

**Gene**	**Primer sequence (5^′^-3^′^, 3^′^-5^′^)**
**ORMDL3**	
5′-3′	CCTCACCAACCTCATTCACAAC
3′-5′	TACAGCACGATGGGTGTGATG
**GAPDH**	
5′-3′	TGACTTCAACAGCGACACCCA
3′-5′	CACCCTGTTGCTGTAGCCAAA
**MMP-9**	
5′-3′	GCTGGGCTTAGATCATTCCT
3′-5′	CATTCACGTCGTCCTTATGC
**VEGF**	
5′-3′	ACAGGGATGAGGACACCG
3′-5′	GGGCTGCTTCTTCCAACA

### Tube Formation Assay on ORMDL3

Human umbilical vein endothelial cells (HUVECs) were incubated in the serum starvation condition (1% FBS) for 24 h. Cells were seeded in a Matrigel-coated, 96-well microplate (10,000 cells/well). After incubation (4 h) to allow them to form blood vessel-like networks, cells were incubated for an hour at 37°C. The images were analyzed by scanning with CQ1 instrument.

### Statistical Analysis

Statistical analysis was performed using SPSS 20.0 (IBM). All data were expressed as mean ± standard deviation (mean ± SD). Kruskal–Wallis and one-way analysis of variance (ANOVA) were used to analyze the statistical differences among multiple groups. Pearson correlation analysis was used to analyze the correlation. *P*-value < 0.05 was set at statistical significance level.

## Results

### Airway Angiogenesis Aggravated in Asthma

In the asthmatic group, tracheal epithelial cells were shed, a large number of lymphocytes and macrophages had infiltrated into the bronchial walls, and the smooth muscle and bronchial epithelial layers were thickened (Figures 1A–C). There were no signs of epithelial cell proliferation or inflammatory infiltration index (mean average: 6.23) in the lungs of healthy control mice. In the budesonide-treated group, peribronchial inflammation cells were significantly reduced (score in HE staining, mean average: 17.73) compared with the asthmatic group (mean average: 27.05, *P* < 0.01), while not entirely ameliorated to the control level (*H*-value = 26.801, *P* < 0.01).

**Figure 1:** Airway angiogenesis aggravated in asthma. **(A–C)** Bronchial hyperplasia in asthma (HE staining). **(A)** The asthmatic group, **(B)** the budesonide-treated group, **(C)** the normal control group. Magnification, ×400. Bronchial hyperplasia was observed using HE staining. **(A)** Damaged tracheal structures and infiltration of the inflammatory cells were observed in the asthmatic group (mean rank: 27.05). **(B)** Damaged tracheal structures and infiltration of inflammatory cells were alleviated in the budesonide-treated group (mean rank: 17.73). **(C)** Relatively complete bronchial structures were in the normal control group (mean rank: 6.23). **(D–F)** Increased collagen deposition in asthma using Masson staining. **(D)** The asthmatic group, **(E)** the budesonide-treated group, **(F)** the normal control group. Magnification, ×400. Increased collagen deposition in lung tissues was determined using Masson staining. **(D)** Substantial collagen deposition was observed in the interstitium of the asthmatic mice (mean rank: 19.83). **(E)** Collagen deposition was reduced in the budesonide-treated group (mean rank: 15.67). **(F)** Little collagen deposition in interstitium was observed in the control group (mean rank: 6.50). **(G–J)** Expression of CD31 in lung tissues. **(G)** The asthmatic group, **(H)** the budesonide-treated group, **(I)** the normal control group. Magnification, ×200. **(J)** CD31 intensity in lung tissues. Expression of CD31 protein in lung tissues was investigated using immunohistochemistry. Vessel area was increased in the asthmatic group compared with that in the control group and decreased in the budesonide- treated group. *P < 0.01, the asthmatic group vs. the normal control group. ^#^*P* < 0.01 the asthmatic group vs. the budesonide-treated group. ^▴^*P* < 0.01, the budesonide-treated group vs. the normal control group.

The airway walls were thin, and mucosal structures were intact without obvious smooth muscle hyperplasia or collagen deposition in the control group. In the asthmatic group, large deposits of collagen surrounded the vessels and alveolar interstitium (Figures 1D–F), and the collagen-staining index (mean average: 19.83) was significantly higher compared with the control group (mean average: 6.50). After budesonide treatment, the collagen deposition (mean average: 15.67) was significantly reduced compared with the asthmatic group although still higher than the control group (*H*-value = 14.981, *P* < 0.01).

The endothelial cell surface was marked with CD31 (12). The CD31 expression level of lung tissues was detected by immunohistochemical staining. Obviously, CD31 expression increased in the asthmatic group compared with that in the control group (21.695 ± 3.89 vs. 10.183 ± 2.89%, *P* < 0.01). Administration of budesonide significantly reduced CD31 expression compared with that in the asthmatic group (17.775 ± 2.10 vs. 21.695 ± 3.89%, *P* < 0.01) although it did not entirely reduce to the control levels (17.775 ± 2.10 vs. 10.183 ± 2.89%, *P* < 0.01). The levels of CD31 staining were quantified using Image J software (Figures 1G–J). Our results demonstrate the upregulation of angiogenesis in asthma.

### ORMDL3, p-ERK1/2, VEGF, and MMP-9 Expression Increased in Asthmatic Mice

The ORMDL3 expression level of lung tissues was detected by immunohistochemical staining. ORMDL3 expression was significantly increased in the asthmatic group (Figures 2A–C) compared with that in the control group (55.81 ± 5.45 vs. 11.07 ± 4.51%, *P* < 0.01). Administration of budesonide significantly reduced ORMDL3 expression compared with that in the asthmatic group (31.43 ± 3.62 vs. 55.81 ± 5.45%, *P* < 0.01), but it did not entirely reduce to the control level (31.43 ± 3.62 vs. 11.07 ± 4.51%, *P* < 0.01). The ORMDL3 levels were quantified using Image J software (Figure 2D). These observations were confirmed by Western blotting: ORMDL3 protein was increased in asthmatic mice compared with the control group (2.77 ± 0.45 vs. 1.25 ± 0.78, *P* < 0.01) and significantly reduced in the budesonide-treated group (2.77 ± 0.45 vs. 1.95 ± 0.74, *P* < 0.05, *P* = 0.011, Figure 2E) without returning to the normal level.

**Figure 2:** Expression of ORMDL3, p-ERK1/2 increased in asthmatic mice. **(A–E)** Expression of ORMDL3 in lung tissues. **(A)** The asthmatic group, **(B)** the budesonide-treated group, **(C)** the control group. Magnification, ×200. **(D)** ORMDL3 protein expression quantified with Image J. **(E)** ORMDL3 expression with Western blotting. ORMDL3 expression in lung tissues was investigated using immunohistochemistry **(A–D)**. ORMDL3 was increased in the asthmatic group and decreased in the budesonide-treated group compared with that in the normal control group. *P < 0.01, the asthmatic group vs. the control group. ^#^*P* < 0.01, the asthmatic group vs. the budesonide-treated group. ^▴^*P* < 0.01, the budesonide-treated group vs. the control group. **(F–J)** Expression of p-ERK in lung tissues **(F)** The asthmatic group, **(G)** the budesonide-treated group, **(H)** the control group. Magnification, ×200. **(I)** p-ERK protein expression was quantified with Image J. **(J)** p-ERK expression with Western blotting. Expression of p-ERK protein in lung tissues was investigated using immunohistochemistry **(F–I)**. p-ERK expression was increased in the asthmatic group compared with that in the control group and decreased in the budesonide-treated group. *P < 0.01, the asthmatic group vs. the normal control group; ^#^*P* < 0.01, the asthmatic group vs. the budesonide-treated group; ^▴^*P* < 0.01, the budesonide-treated group vs. the normal control group.

The p-ERK1/2 expression level of lung tissues was detected by immunohistochemical staining. A low level of p-ERK1/2 expression was detected in the control group, which was increased in the asthmatic group (14.64 ± 3.66 vs. 50.89% ± 9.91%, *P* < 0.01) by immunohistochemical staining (Figures 2F–I). Administration of budesonide significantly reduced p-ERK1/2 expression (30.17 ± 3.00 vs. 50.89 ± 9.91%, *P* < 0.01), still above the control level (30.17 ± 3.00 vs. 14.64 ± 3.66%, *P* < 0.01). A similar result was confirmed by Western blotting (Figure 2J); p-ERK1/2 protein was increased in asthmatic mice compared with the control group (16.11 ± 4.92 vs. 7.83 ± 2.27, *P* < 0.01) and significantly reduced by administration of budesonide (16.11 ± 4.92 vs. 12.07 ± 3.44, *P* < 0.05, *P* = 0.022; Figure 2H) without reaching the normal standard.

The VEGF expression level of lung tissues was detected by immunohistochemical staining. Vascular endothelial growth factor expression was increased in the asthma group (Figures 3A–D) compared with that in the control group (26.84 ± 2.46 vs. 9.92 ± 2.79%, *P* < 0.01) by immunohistochemical staining. A low level of VEGF expression was detected in the control group. Budesonide ameliorated VEGF expression compared with the asthmatic group (17.46 ± 2.03 vs. 26.84 ± 2.46%, *P* < 0.01) but above the control level (17.46 ± 2.03 vs. 9.92 ± 2.79%, *P* < 0.01).

**Figure 3:** VEGF, MMP-9 expression increased in asthmatic mice. **(A–D)** Expression of VEGF in lung tissues. **(A)** The asthmatic group, **(B)** the budesonide-treated group, **(C)** the control group. Magnification ×200. **(D)** VEGF protein expression quantified with Image J. Expression of VEGF in lung tissues was investigated using immunohistochemistry **(A–D)**. VEGF expression was increased in the asthmatic group compared with that in the normal control group and decreased in the budesonide-treated group. *P < 0.01, the asthmatic group vs. the normal control group, ^#^*P* < 0.01, the asthmatic group vs. the budesonide-treated group, ^▴^*P* < 0.01, the budesonide-treated group vs. the normal control group. **(E–I)** Expression of MMP-9 in lung tissues. **(E)** The asthmatic group, **(F)** the budesonide-treated group, **(G)** the normal control group. Magnification, ×200. **(H)** MMP-9 protein expression quantified with Image J. **(I)** Western blotting expression of MMP-9. Expression of MMP-9 in lung tissues was investigated using immunohistochemistry **(E–H)**. MMP-9 expression was increased in the asthmatic group compared with that in the control group and decreased in the budesonide-treated group. *P < 0.01, the asthmatic group vs. the control group, ^#^*P* < 0.01, the asthmatic group vs. the budesonide-treated group, ^▴^*P* < 0.01, the budesonide-treated group vs. the control group.

The MMP-9 expression level of lung tissues was detected by immunohistochemical staining. MMP-9 levels were obviously increased in the asthmatic group compared with that of the control group (Figures 3E–H) (44.29 ± 6.17 vs. 14.87 ± 3.85%, *P* < 0.01). It is worth mentioning that MMP-9 expression was significantly ameliorated with budesonide treatment (24.71 ± 3.95 vs. 44.29 ± 6.17%, *P* < 0.01), but it was not reduced to the control level (44.29 ± 6.17 vs. 14.87 ± 3.85%, *P* < 0.01). Western blotting confirmed the observation (Figure 3I). The level of MMP-9 protein was increased in asthmatic mice compared with the control group (2.69 ± 1.08 vs. 0.72 ± 0.58, *P* < 0.01) and significantly reduced by administration of budesonide (2.69 ± 1.08 vs. 1.59 ± 0.83, *P* < 0.05, *P* = 0.007) without reaching the control level.

### ORMDL3 Expression Associated With Angiogenesis in Asthma

Results show that ORMDL3 levels, detected by immunohistochemical staining, were significantly positively associated with CD31 (*r* = 0.661, *P* < 0.01), p-ERK (*r* = 0.731, *P* < 0.01), and VEGF (*r* = 0.854, *P* < 0.01). There was a positive association between VEGF and p-ERK1/2 (*r* = 0.676, *P* < 0.01). As marker CD31 is a characteristic feature of angiogenesis, these data indicate that ORMDL3 may serve a key role in vessel remodeling.

### Infection of BEAS-2B Cells With ORMDL3-Overexpressed Lentiviral Vector

After infecting the ORMDL3-overexpressed lentiviral vector into BEAS-2B cells, green fluorescent protein expression using fluorescence rate (80%) confirmed the successful infection (Figures 4A–D). The quantitative PCR results showed that the ORMDL3 gene expression in the OE group was 2.658 times that in the control (NC) group (*P* = 0.0000) (Figure 4E). Thus, the lentiviral vector overexpressing ORMDL3 effectively infected BEAS-2B cells.

**Figure 4:** Infection of the recombinant lentiviral vector into BEAS-2B cells. The plasmids were introduced into BEAS-2B cells, the lentiviral vector overexpressing ORMDL3 was successfully constructed and effectively infected BEAS-2B cells. Fluorescence rate was the positive infection rate **(A–D)**. OE **(B,D)**: the group infected with the lentiviral vector overexpressing ORMDL3 NC **(A,C)**: the normal group. Magnification, ×200 (B is bright field, G is the fluorescence field). **(E–G)** ORMDL3, VEGF, and MMP-9 mRNA expression in ORMDL3-overexpressed BEAS-2B cells. In the infected BEAS-2B cells with the ORMDL3-overexpressed lentiviral vector, the mRNA expressions of angiogenesis biomarkers (VEGF/MMP-9) were increased compared with that in the control group. The quantitative PCR results show that the ORMDL3 gene expression in the OE group was 2.658 times that in the NC group (*P* = 0.0000) **(E)**; the VEGF expression in the OE group was 2.036 times that in the NC group (*P* = 0.000366182) **(F)**; MMP-9 gene expression in the OE group was 1.443 times that in NC group (*P* = 0.035845639) **(G)**. **(H–J)** VEGF, MMP-9, and ORMDL3 protein expression in ORMDL3-overexpressed BEAS-2B cells. **(H)** ORMDL3 expression, **(I)** MMP-9 expression, **(J)** VEGF expression. In the infected BEAS-2B cells with the ORMDL3-overexpressing lentiviral vector, the protein expressions of ORMDL3 and angiogenesis biomarkers (VEGF/MMP-9) were progressively increased compared with that in the control group. **(K–N)** Tube formation assay. **(K)** Negative control, **(L)** NC, the negative-infected group; **(M)** PC, positive control; **(N)** OE, the positive infected group with the ORMDL3-overexpressing lentivirus. Magnification, ×200. There is no difference between the NC and OE groups.

### ORMDL3 Induced MMP-9 and VEGF Expression

After successful infection in the BEAS-2B cells, the quantitative PCR results show that the VEGF gene expression in the OE group was 2.036 times that in the NC group (*P* = 0.000366182) (Figure 4F), and the MMP-9 gene expression in the OE group was 1.443 times that in the NC group (*P* = 0.035845639) (Figure 4G). Western blotting confirmed the observation. The level of ORMDL3 protein was increased in the OE group compared with the NC group (0.6117 ± 0.010 vs. 0.037 ± 0.001, *P* < 0.01) (Figure 4H). The level of MMP-9 protein was increased in the OE group compared with the NC group (0.077 ± 0.011 vs. 0.046 ± 0.009, *P* < 0.05, *P* = 0.019) (Figure 4I). The level of VEGF protein was as well (1.272 ± 0.049 vs. 1.028 ± 0.034, *P* < 0.01, *P* = 0.002) (Figure 4J). The increase of these angiogenesis biomarkers indicates that ORMDL3 activates expression of VEGF and MMP-9 and vessel formation.

### Tube Formation Assay

After successful infection of ORMDL3 overexpressing lentiviral vector to HUVECs, tube formation was analyzed by the CQ1 instrument. These results show that the vessel junction and length in the OE group was similar to that in the control (NC) group (*P* >0.05, *P* = 0.6329, *P* = 0.6330) (Figures 4K–N). Successful infection of ORMDL3 overexpressing lentiviral vector to HUVECs does not influence neovascularization.

## Discussion

Our studies in OVA-induced mice show CD31 and ORMDL3 were significantly upregulated in asthma. CD31 is widely used in evaluating the increase of size and number of blood vessels. The increases of size and number of blood vessels as well as vascular leakage are associated with structural changes of the airway wall in asthma (11). Angiogenesis is the hallmark feature in asthmatic airway remodeling. There is a positive correlation between ORMDL3 and endothelial marker-CD31, suggesting a role of ORMDL3 in the formation of new blood vessels in asthma. ORMDL3 significantly contributed to the development of angiogenesis; it can be regarded as an indicator of angiogenesis in asthma. Administration of budesonide significantly reduced angiogenesis and ORMDL3 expression; these findings were consistent with previous studies (8, 9), and the mechanism of asthmatic angiogenesis needs to be further clarified. A tube formation assay *in vitro* is to be completed to examine the effect of ORMDL3 on angiogenesis. However, successful infection of ORMDL3 overexpressing lentiviral vector to HUVECs do not influence neovascularization. Faiz A found that angiogenic regulatory influence of extracellular matrix (ECM) deposited by asthma is similar to non-asthmatic airway smooth muscle cells in the resting state (12). We found that MMP-9 and VEGF had upregulated in BEAS-2B cells infected with ORMDL3-overexpressing vectors. However, the tube formation assay was negative. Only the effects of cytokines from culture medium supernatant had been added to HUVECs. In fact, when ORMDL3-overexpressioning plasmid infected bronchial epithelial cells promoted the expression of VEGF and MMP9, only a small part was secreted into the culture medium supernatant for the tube formation assay. It needs further experimentation to confirm the total angiogenesis effects. Vascular endothelial growth factor is a potent inducer of vascular permeability. Vascular endothelial growth factor plays an integral role in regulating vascular barrier function physiologically and in pathologies, including cancer, stroke, cardiovascular disease, retinal conditions, and asthma (3, 13). In a hypoxia environment, VEGF binds to VEGF receptors on the endothelial cell membrane and causes self-phosphorylation of the receptor. The role of VEGF is to take effect *in vivo*. In ameliorated-regulatory effects of budesonide on the hypoxia environment *in vivo*, CD31 and ORMDL3 expression were decreased in lung tissues of the budesonide-treated mice, compared with that in asthmatic mice (14). Therefore, there is no hypoxia and inflammation environment, and the effect ORMDL3 on the tube formation assay *in vitro* is little.

Many studies demonstrate that increased hypervascularity of bronchial wall cells closely pertain to the expression of angiogenic factors, such as MMP-9 and VEGF. During the process of angiogenesis, the ECM is degraded by MMPs in progression to facilitate endothelial cell invasion and lead to sprouting of new vessels (14, 15). The roles of MMP-9 in angiogenesis include the release of VEGF and/or basic fibroblast growth factor (FGF-2) (16). At the same time, VEGF also strongly stimulates MMP-9 production and allergic inflammation (17, 18). Furthermore, as an “angiogenic switch,” VEGF is reported to induce vascular leakage, vessel permeability, and angiogenesis. As a driver of airway angiogenesis, VEGF induces cell migration and transformation of endothelial cells. In our animal experiment, it was found that MMP-9 and VEGF expression were significantly upregulated in asthmatic mice. Further in our *in vitro* experiment, after successful infection of ORMDL3 overexpressing lentiviral vector to BEAS-2B cells, MMP-9 and VEGF levels were significant increased, which indicated that ORMDL3 induced MMP-9 and VEGF expression. Positive correlation was further found between the ORMDL3 and p-ERK1/2, VEGF, also between p-ERK1/2 and VEGF. Our results demonstrate that ORMDL3 contributes to angiogenesis, increasing VEGF/MMP-9 expression possibly through the ERK1/2 pathway. OrMDL3 can bind and inhibit sarcoplasmic reticulum calcium ATPase activity and increase unfolded protein response (UPR). Unfolded protein response is a group of intracellular signal transduction pathways (IRE1, p-ERK, ATF6). p-ERK plays an important role in the UPR. It is worth noting that the p-ERK/eIF2α/ATF4 pathway was found to activate VEGF expression in human vascular endothelial cells. p-ERK was indicated to be the intermediate link of ORMDL3 with angiogenic factors, such as VEGF (19, 20).

The study on the mechanism of angiogenesis in asthma is beneficial for not only understanding of airway remodeling, but also providing a potential therapeutic target. In the development of inhibiting MMPs (MMP-2, MMP-9, and MT1-MMP), selective MMP inhibitors have included unique modes of action implicated in angiogenesis (3, 21, 22). Pancreatic cancer patients are reported to get significantly improved survival though application of MMP inhibitor (marimostat) in combination with gemcitabine. In a mouse model of breast cancer, presurgical treatment with an oral MMP inhibitor even improved survival from 67 to 92% (23). However, MMP-9 deficiency in mouse models led to increased interleukin-6 levels in the bone marrow, which promoted pancreatic ductal adenocarcinoma (PDAC) invasion and metastasis. Furthermore, VEGF may also serve as an driver because it can lead to upregulation of other pro-angiogenic factors (24). Vascular endothelial growth factor and MMP-9 are shown to be a key target in the “angiogenic on-off.”

In general, we illustrate the association between ORMDL3 and angiogenic factors, such as MMP-9 and VEGF in asthma. During this process, ORMDL3 induces the upregulation of MMP-9 and VEGF, and contributes to the airway angiogenesis and asthmatic airway remodeling. Counting on these results, we might offer a possible therapeutic target for preventing asthmatic angiogenesis. Further research is needed to confirm this conclusion.

## Data Availability Statement

The original contributions presented in the study are included in the article/supplementary materials, further inquiries can be directed to the corresponding author/s.

## Ethics Statement

The animal study was reviewed and approved by Ethics Committee of Shandong University. Written informed consent was obtained from the owners for the participation of their animals in this study.

## Author Contributions

All authors listed have made a substantial, direct, and intellectual contribution to the work and approved it for publication.

## Funding

This study was supported by the Shandong Provincial Natural Science Foundation (grant no. ZR2020MH003).

## Conflict of Interest

The authors declare that the research was conducted in the absence of any commercial or financial relationships that could be construed as a potential conflict of interest.

## Publisher's Note

All claims expressed in this article are solely those of the authors and do not necessarily represent those of their affiliated organizations, or those of the publisher, the editors and the reviewers. Any product that may be evaluated in this article, or claim that may be made by its manufacturer, is not guaranteed or endorsed by the publisher.

## References

[1] ClarkeTCNorrisTSchillerJS. Early Release of Selected Estimates Based on Data from the 2016 National Health Interview Survey. Hyattsville, MA: National Center for Health Statistics (2016).

[2] ParkSYKimJHKimHJSeoBKwonOYChangHS. High prevalence of asthma in elderly women: findings from a Korean national health database and adult asthma cohort. Allergy Asthma Immunol Res. (2018) 10:387–96. 10.4168/aair.2018.10.4.38729949835PMC6021593

[3] BolandiSMAbdolmalekiZAssarehzadeganMA. Anti-angiogenic properties of bevacizumab improve respiratory system inflammation in ovalbumin-induced rat model of asthma. Inflammation. (2021) 44:2463–75. 10.1007/S10753-021-01516-W34420156PMC8380193

[4] MoffattMFKabeschMLiangLDixonALStrachanDHeathS. Genetic variants regulating ORMDL3 expression contribute to the risk of childhood asthma. Nature. (2007) 448:470–3. 10.1038/nature0601417611496

[5] MillerMTamABChoJYDohertyTAPhamAKhorramN. ORMDL3 is an inducible lung epithelial gene regulating metalloproteases, chemokines, OAS, and ATF6. Proc Natl Acad Sci USA. (2012)109:16648–53. 10.1073/pnas.120415110923011799PMC3478632

[6] LeeKSMinKHKimSRParkSJParkHSJinGY. Vascular endothelial growth factor modulates matrix metalloproteinase-9 expression in asthma. Am J Respir Crit Care Med. (2006) 174:161–70. 10.1164/rccm.200510-1558OC16645174

[7] FelsenCNSavariarENWhitneyMTsienRY. Detection and monitoring of localized matrix metalloproteinase upregulation in a murine model of asthma. Am J Physiol Lung Cell Mol Physiol. (2014) 306:L764–74. 10.1152/ajplung.00371.201324508733PMC3989727

[8] YuFSunYYuJDingZWangJZhangL. ORMDL3 is associated with airway remodeling in asthma via the ERK/MMP-9 pathway. Mol Med Rep. (2017) 15:2969–76. 10.3892/mmr.2017.641328358425PMC5428751

[9] SunYWangJLiHSunLWangYHanX. The effects of budesonide on angiogenesis in a murine asthma model. Arch Med Sci. (2013) 9:361–7. 10.5114/aoms.2013.3319423671450PMC3648823

[10] ZhangCZhangLHWuYFLaiTWWangHSXiaoH. Suhuang antitussive capsule at lower doses attenuates airway hyperresponsiveness, inflammation, and remodeling in a murine model of chronic asthma. Sci Rep. (2016) 6:21515. 10.1038/srep2151526861679PMC4748281

[11] ChenYCSheuJJChiangJYShaoPLWuSCSungPH. Circulatory rejuvenated EPCs derived from PAOD patients treated by CD34^+^ cells and hyperbaric oxygen therapy salvaged the nude mouse limb against critical ischemia. Int J Mol Sci. (2020) 21:7887. 10.3390/ijms2121788733114267PMC7660611

[12] FaizAHarknessLMTjinGBernalVHorvatovichPJamesA. Angiogenic regulatory influence of extracellular matrix deposited by resting state asthmatic and non-asthmatic airway smooth muscle cells is similar. J Cell Mol Med. (2021) 25:6438–47. 10.1111/jcmm.1664834146379PMC8256353

[13] MeyerNAkdisCA. Vascular endothelial growth factor as a key inducer of angiogenesis in the asthmatic airways. Curr Allergy Asthma Rep. (2013) 13:1–9. 10.1007/s11882-012-0317-923076420

[14] ZouLPZhangXZhangYXuXJWangTF. Down-regulatory effects of budesonide on expression of STAT6 and ORMDL3 in lung tissues of asthma mice. Zhongguo Dang Dai Er Ke Za Zhi. (2014) 16:198–202. 10.7499/j.issn.1008-8830.2014.02.02124568918

[15] Soltanpour GharibdoustiFFazeli DelshadBFalakRShayanfarNGanjalikhani HakemiMAndalibA. Induction of humoral immune responses and inhibition of metastasis in mice by a VEGF peptide-based vaccine. Iran J Basic Med Sci. (2020) 23:507–14. 10.22038/ijbms.2020.38508.914132489566PMC7239427

[16] ShibuyaM. Tyrosine kinase receptor Flt/VEGFR family: its characterization related to angiogenesis and cancer. Genes Cancer. (2010) 1: 1119–23. 10.1177/194760191039298721779435PMC3092272

[17] KangHHongZZhongMKlompJBaylessKJMehtaD. Piezo1 mediates angiogenesis through activation of MT1-MMP signaling. Am J Physiol Cell Physiol. (2019) 316:C92–103. 10.1152/ajpcell.00346.201830427721PMC6383143

[18] YangLZhangLHuJWangWLiuX. Promote anti-inflammatory and angiogenesis using a hyaluronic acid-based hydrogel with miRNA-laden nanoparticles for chronic diabetic wound treatment. Int J Biol Macromol. (2021) 166:166–78. 10.1016/J.IJBIOMAC.2020.10.12933172616

[19] KimEJLeeHLeeYJSonnJKLimYB. Ionizing radiation regulates vascular endothelial growth factor-a transcription in cultured human vascular endothelial cells via the PERK/eIF2α/ATF4 pathway. Int J Radiat Oncol Biol Phys. (2020) 107:563–70. 10.1016/j.ijrobp.2020.03.00332169411

[20] ChenJMillerMUnnoHRosenthalPSandersonMJBroideDH. Orosomucoid-like 3 (ORMDL3) upregulates airway smooth muscle proliferation, contraction, and Ca^2+^ oscillations in asthma. J Allergy Clin Immunol. (2018) 142:207–18.e6. 10.1016/j.jaci.2017.08.01528889952PMC5842097

[21] WinerAJanoskyMHarrisonBZhongJMoussaiDSiyahP. Inhibition of breast cancer metastasis by presurgical treatment with an oral matrix metalloproteinase inhibitor: a preclinical proof-of-principle study. Mol Cancer Ther. (2016) 15:2370–7. 10.1158/1535-7163.MCT-16-019427466357PMC5050118

[22] FieldsGB. Mechanisms of actaion of novel drugs targeting angiogenesis-promoting matrix metalloproteinases. Front Immunol. (2019) 10:1278. 10.3389/FIMMU.2019.0127831214203PMC6558196

[23] PałganKBartuziZ. Angiogenesis in bronchial asthma. Int J Immunopathol Pharmacol. (2015) 28:415–20. 10.1177/039463201558090725875602

[24] BajboujKRamakrishnanRKHamidQ. Role of matrix metalloproteinases in angiogenesis and its implications in asthma. J Immunol Res. (2021) 2021:6645072. 10.1155/2021/664507233628848PMC7896871

